# Different Dual-Task Paradigm Reduce Postural Control Ability and Dynamic Stability of Healthy Young Adults during Stair Descent

**DOI:** 10.1155/2024/9942042

**Published:** 2024-03-11

**Authors:** Jiankang Yang, Shifang Yan, Chuanbao Cao

**Affiliations:** ^1^Department of Physical Education, College of Sports and Arts, Dong-A University, Busan 49315, Republic of Korea; ^2^Department of Wushu, Hebei Sport University, Shijiazhuang 050000, Hebei, China

## Abstract

**Objective:**

This study aimed to compare the impacts of different dual-task paradigms on the postural control ability and dynamic stability of the youth during stair descent.

**Method:**

Twenty young adults without regular exercise habits were randomly recruited to perform stair descent tasks with three different paradigms: single-task, cognitive dual-task, and manual dual-task. Kinematic and dynamic data were collected using an 8 Vicon motion analysis system and a Kistler force plate to evaluate postural control ability and dynamic stability during stair descent.

**Results:**

The variation trends of lower limb joint moment were similar under the three task models. Compared with a single-task, both dual-task paradigms significantly reduced the mechanical parameters and dynamic stability during stair descent.

**Conclusion:**

The dual-task paradigm increases the risk of stair-related falls. Both cognitive and manual tasks have similar impacts on postural control ability and dynamic stability during stair walking. It is recommended that people avoid performing dual tasks during stair descent.

## 1. Introduction

Stair negotiation is one of the most challenging daily activities. When walking on stairs, the risk of falls during stair descent is three times higher than during stair ascent [1]. Stair walking, compared to level walking, demands greater joint moment and range of motion in the lower limbs, resulting in higher “functional consumption” [2, 3]. Abnormal gait has been identified as the primary cause of falls during stair negotiation [4]. During stair descent, the toes initially make contact with the ground, and the peak of the ground reaction force (GRF) occurs earlier [5], indicating decreased stability and a significantly increased risk of falls.

Stair negotiation often involves mental or physical tasks alongside physical activity. In dual-task (DT) conditions, compared to single-task (ST), distractions occur [6], affecting the information integration and motion control abilities of the human system, leading to reduced postural control [7]. Pellecchia [8] found that performing cognitive tasks (CT) during stair descent significantly increases the velocity of the body's centre of mass (COM) and raises the risk of falls. Research by Madehkhaksar and others suggests that manual tasks (MT), similar to CT, also negatively affect stair negotiation. MT interference reduces walking velocity while increasing the amplitude of the plantar centre of pressure (COP) [9]. It is widely acknowledged that human postural control ability diminishes when performing DT [8]. However, the distinction between CT and MT in influencing body stability during stair descent remains unclear [9, 10].

Previous studies have mainly used traditional static stability theory to assess physical stability during stair walking [2, 3, 6]. This theory primarily examines the relationship between the projection of the COM onto the sagittal and frontal planes [6] or considers the velocity and amplitude of COM and COP [2]. However, stair negotiation is a dynamic activity, and it is necessary to consider how both COM velocity and position influence dynamic stability [11]. Following dynamic stability theory, Zheng et al. [11] defined the COM influenced by velocity as the extrapolated COM and its minimum distance to the boundary of the supporting surface as the margin of stability (MOS). While MOS has been applied in walking and running research, it is rarely used to assess stability during stair negotiation [12–14].

This study aimed to explore the difference between CT and MT paradigms in influencing human postural control and dynamic stability during stair descent so as to enrich the theory of fall prevention during stair negotiation. In this study, it was hypothesised that (1) DT interference may significantly reduce the mechanical parameters and dynamic stability during stair descent and (2) CT interference has a greater impact on physical stability during stair descent than MT interference.

## 2. Materials and Methods

### 2.1. Participants

The required sample size was calculated using the G^*∗*^Power Version, referencing a relevant study [15]. The power was set to 0.8, *α* to 0.05, the effect size to 0.4, and the number of groups to 2. The sample size required for a single group was calculated as 19. Twenty subjects meeting the screening criteria were randomly recruited. Inclusion criteria were as follows: age between 20 and 30 years, no regular exercise habits, and no history of falls in the past 6 months. Exclusion criteria included musculoskeletal diseases and visual and vestibular dysfunctions affecting postural control ability. Ultimately, 20 young subjects were selected (age: 24.6 ± 3.2 years; body height: 162.5 ± 4.6 cm; body weight: 57.6 ± 6.5 kg; BMI: 22.3 ± 2.5). All subjects were informed about the experimental procedures and potential risks and provided written informed consent. This study was approved by the internal review board of Hebei Sport University and conducted in accordance with the Declaration of Helsinki.

### 2.2. Equipment and Data Collection

An iron staircase with six steps was used to simulate the use of stairs in daily life. The staircase weighed about 1.5 tons, effectively reducing the resonance between the staircase and the force plate. The step dimensions were 0.3 m tread × 1.5 m width × 0.17 m riser, with an inclination angle of 29.4°. Kinematic data were collected using an eight-camera motion analysis system (Vicon Motion System, UK) and matched infrared reflective markers (*d* = 14 mm, UK) at a sampling rate of 100 Hz. Dynamic data were collected by a Kistler force plate (Kistler 9287BA, Winterthur, Switzerland), which was embedded in the groove of the third step of the staircase, with a GRF of 1,000 Hz.

### 2.3. Procedures

The subjects were required to wear uniform clothes and shoes for body morphology measurement and dominant leg test. According to the test, all the subjects were right-side dominant. The marks were pasted on the bony landmarks of the subjects. In the formal trial, the subjects were instructed to walk down the stairs in a step-by-step manner under ST, CT, and MT conditions, respectively. In this study, under ST, the subjects only walked on the stairs without additional motions and tasks. Under the CT, in addition to the stair descent task, the subjects were asked to perform a concurrent task by serially subtracting the value of 3 from the number between 200 and 999 randomly reported by the staff before stair descent [16]. The calculation task ended at the bottom of the staircase. Under MT condition, the subjects were asked to hold a cup filled with water in their right hand during stair descent until the bottom of the staircase [9]. Three valid trials were conducted for each subject.

### 2.4. Data Processing

Raw data were preprocessed using Vicon Nexus 2.5. Then, data files were imported into Visual 3D for filtering, normalisation, and percentage conversion. Kinematic and dynamic data were filtered with a fourth-order Butterworth low-pass digital filter at a cut-off frequency of 6 and 50 Hz, respectively [17]. Step length and step width were calculated from the coordinates of the markers on the subject's heels. The kinematic and dynamic parameters were normalised by time and body weight, respectively. The dominant leg support phase of a step cycle was selected for analysis, and it was defined as the first double support (FDS) phase, single support phase (SSP), and second double support (SDS) phase. FDS was defined as the period from right foot contact with the fourth step to left foot takeoff from the fifth step. SSP began with left foot takeoff from the fifth step to left foot contact with the third step. SDS was defined as the period from left foot contact on the third step and right foot takeoff from the fourth step. Gait velocity was defined as the derivative of the anterior–posterior displacement of human COM to the time [18]. The joint moment was calculated as the flexion and extension moment of the lower limb joints around the frontal axis in the sagittal plane [19]. MOS was defined as the distance between the extrapolated COM and the boundary of the supporting surface [20]. The specific calculation formulas are as follows:

(1) $$\begin{array}{c} \omega_{0}=\sqrt{g/l}, \end{array}$$

(2) $$\begin{array}{c} \text{CM}=D_{\text{COM}}+V_{\text{COM}}/\omega_{0}, \end{array}$$

(3) $$\begin{array}{c} \text{MOS}=B_{\text{MAX}}-\text{CM}, \end{array}$$

where *g* denotes gravitational acceleration, *l* denotes the vertical distance from COM to the ground, and *ω*_0_ denotes the inherent frequency of the inverted pendulum of the human body; *V*_COM_ denotes COM velocity, *D*_COM_ is the COM position of the human body, CM denotes the COM position under the influence of velocity; *B*_MAX_ denotes the maximum value at the boundary of the supporting surface, and MOS denotes dynamic stability. It was found that the most unstable instant of the human body during stair walking is the transient SSP–DSP transition; therefore, it was selected for the comparative analysis of dynamic stability [20, 21].

### 2.5. Statistical Analysis

The averages of three valid data were taken for each subject, and mean ± standard deviation ($\bar{X}\pm \text{SD}$) was used for statistical analysis. Normal distribution and homogeneity tests of dependent variables were carried out with SPSS 20.0. The mechanical parameters and dynamic stability of the subjects during stair descent were compared among the groups using one-way repeated-measures ANOVA. *P* < 0.05 was considered statistically significant.

## 3. Results

### 3.1. Comparison of Dynamic Parameters during Stair Descent under Different DT Conditions

Figure 1 shows that during stair descent, the variations in joint moment in one support phase under the three conditions were consistent but with different peaks. The hip joint moment was dominated by the extension moment in the early stage of the support phase, and about 50% of it was converted into the flexion moment in the support phase, while the flexion moment was dominated in the late stage of the support phase. The knee and ankle joint moments were dominated by extension moment and plantar flexion, respectively.

The positive value of the hip joint moment is the hip joint flexion moment, while the negative value of the hip joint is the hip joint extension moment (Figure 1). The positive value of knee torque is the knee extension moment, while the negative value is the knee flexion moment. The positive value of the ankle moment is the ankle dorsiflexion, while the negative value of the ankle moment is its plantar flexion.

As shown in Table 1, compared with those in ST, the peak hip flexion moment, peak hip extension moment, and second peak knee extension moment during stair descent under DT conditions (CT and MT) decreased in varying degrees, but there were no significant differences (*P* > 0.05). The first peak knee extension moment (*P*=0.031, *P*=0.004, *P*=0.026) and first peak ankle plantar flexion moment (*P*=0.044, *P*=0.027, *P* > 0.05) were significantly higher, while the second peak ankle plantar flexion moment (*P* > 0.05, *P*=0.023, *P* > 0.05) was significantly lower. Compared with that in CT, the first peak knee extension moment under MT was significantly lower (*P*=0.026).

### 3.2. Comparison of Dynamic Stability during Stair Descent under Different DT Conditions

Figure 2 displays the differences in dynamic stability during stair descent under different DT conditions. Results show that compared with those under ST, *D*_COM_ (*P*=0.031, *P*=0.014), *V*_COM_ (*P*=0.001, *P*=0.001), and MOS (*P*=0.001, *P*=0.001) decreased significantly under CT and MT, while *B*_MAX_ showed no significant differences (*P* > 0.05). Compared with the CT interference, *D*_COM_, *V*_COM_, *B*_MAX_, and MOS under MT conditions showed no significant differences (*P* > 0.05).

## 4. Discussion

This study explored the difference in the impact of concurrent CT or MT DT conditions in human postural control and dynamic stability during stair descent. Results showed that DT conditions significantly reduced mechanical parameters and dynamic stability during stair walking, which is consistent with our first hypothesis. Under CT/MT, young adults presented no significant difference in stability during stair descent, which is not in line with our second hypothesis.

Song et al. [22] observed a decrease in the peak torque of lower limb joints under DT conditions. Furthermore, under DT conditions, there was a decrease in the peaks of lower limb joint moments. In line with our results, compared to ST, both CT and MT conditions significantly reduced the peak knee extension moment and plantar flexion moment in subjects during stair descent. This finding lends some support to the hypothesis in this study, which posited that DT would reduce mechanical parameters during stair negotiation. Previous studies have indicated that the mechanical characteristics of lower limb joints play a crucial role in human postural control ability [23]. There is a strong positive correlation between lower limb joint moments and postural control ability [24]. During stair descent, the toes make initial contact with the ground, causing the peak GRF to appear earlier and be more substantial [5]. This necessitates the lower limbs to provide a higher speed and greater damping moment [25]. Inadequate damping velocity or insufficient damping moment can both compromise the stability of the supporting leg and the ability to transition during stair descent, increasing the risk of falls [19]. Our study revealed that dynamic parameters of the lower limbs decreased to varying degrees after DT. Limited attention may be allocated to the secondary task, which might lead to a delay in providing the necessary balance and support for descending stairs promptly. This study suggests that during DTs, to maintain body stability, individuals consciously employ a “soft-landing” self-protection strategy by reducing GRF and lower limb joint moments during stair descent. This reduction in demand for damping velocity and moment aims to decrease the risk of falls.

The dynamic stability of the subjects was significantly reduced under DT conditions. In gait research, dynamic stability pertains to the human body's ability to maintain an upright posture and stability during walking without experiencing falls. MOS is a scientific index used to assess the dynamic stability of the human body. It quantifies the real-time relationship among the supporting surface, COM position, and velocity during motion [20, 26]. A positive MOS indicates a stable state, while a negative MOS suggests an unstable state [20, 26]. Our results revealed that, compared to ST, MOS significantly decreased and became negative under CT and MT conditions, indicating an unstable state of the human body. This finding supports the hypothesis of this study. Madehkhaksar's study has shown that MT can lead to a decrease in step speed and a significant increase in the amplitude of medial and lateral COM during stair descent, affecting the body's stability during stair walking [9]. The results of our study indicated that compared to ST interference, both MT and CT paradigms led to a significant reduction in COM velocity during stair descent. This aligns with previous research indicating that performing dual tasks results in decreased step speed [8, 27]. Hamel and Cavanagh [27] proposed that individuals actively employ a “conservative” strategy of slowing down during DT performance, and the reduction in COM velocity helps control body movement more effectively to minimise the risk of falls. It has been observed that the boundary of the supporting surface is a significant factor affecting MOS during stair negotiation, and increasing the supporting surface can improve MOS [20, 28]. In our study, we observed a trend of increased supporting surface boundaries in the DT model, although the difference was not statistically significant. This trend may be due to expanding the supporting plane to enhance physical stability and consequently reduce the risk of falls.

CT/MT had the same impact on the dynamic stability of young adults during stair descent. The “capacity sharing model” theory of O'Shea et al. [29] pointed out that DTs have higher requirements for attention and executive force, and performing a dual-task paradigm simultaneously will lead to a decline in the performance of both tasks or one of them. This study revealed that compared with the ST interference, the subjects' gait velocity, lower limb dynamic parameters, and MOS decreased to varying degrees during stair descent under DT conditions (CT and MT). Limited attention may be allocated to the second task, potentially leading to a delay in promptly providing the necessary balance and support for descending stairs. Limited attention may be allocated to the second task and be unable to quickly provide damping and supporting moments for stair descent, presenting an unstable state. Therefore, the addition of the second task negatively affected the dynamic stability of the human body during stair descent. Furthermore, compared with CT, in addition to reducing the first peak knee extension moment, MT had no significant differences in other mechanical parameters or dynamic stability. A previous study found that both CT and MT executions are controlled by cerebral nerves [30]. MT execution is not an unconscious neuromuscular control and requires attention resources and spatial cognitive resources from the brain [31]. This may be the reason why the two DTs have similar impacts on the human body during stair negotiation.

## 5. Conclusions

Compared with ST, the subjects presented with a lower COM velocity, reduced peaks of knee extension moment and plantar flexion moment, and decreased dynamic stability during stair descent under both CT and MT. DT has a significantly negative impact on the dynamic stability of the human body during stair descent. To maintain body stability, the human body adopts a self-protection strategy to reduce the COM velocity and GRF during stair descent. Both CT and MT have similar impacts on gait parameters, postural control ability, and dynamic stability. Therefore, other tasks should be avoided during stair negotiation. If it is necessary to perform multiple tasks, reducing the COM velocity is a more scientific strategy during stair negotiation.

## Figures and Tables

**Figure 1:** Time-varying curves of hip, knee, and ankle joint moment.

**Figure 2:** Comparison results of dynamic stability during stair descent under different DT conditions. *Notes*: a, significantly different compared with ST after interference with this task; ST, single task; CT, cognitive task; MT, manual task.

**Table 1:** Comparison of mechanical parameters of the lower limbs.

	ST	CT	MT
Peak hip flexion moment (N · m/kg)	0.34 ± 0.11	0.28 ± 0.04	0.25 ± 0.04
Peak hip extension moment (N · m/kg)	−0.38 ± 0.14	−0.40 ± 0.12	−0.34 ± 0.08
First peak knee extension moment (N · m/kg)	0.92 ± 0.14	0.77 ± 0.13^a^	0.54 ± 0.10^ab^
Second peak knee extension moment (N · m/kg)	1.27 ± 0.17	1.33 ± 0.11	1.16 ± 0.14
First peak ankle plantar flexion moment (N · m/kg)	−1.14 ± 0.16	−0.99 ± 0.20^a^	−0.94 ± 0.13^a^
Second peak ankle plantar flexion moment (N · m/kg)	0.76 ± 0.10	0.80 ± 0.12^a^	0.89 ± 0.16

*Notes*: ^a^Significantly different compared with ST after interference with this task; ^b^significant difference between CT and MT. ST, single task; CT, cognitive task; MT, manual task.

## Data Availability

The data used to support the findings of this study are available from the corresponding author upon request.
